# The Influence of Air Pollution on Pulmonary Disease Incidence Analyzed Based on Grey Correlation Analysis

This article has been retracted.

**DOI:** 10.1155/2022/4764720

**Published:** 2022-09-30

**Authors:** Yujiao Jiao, Cuike Gong, Shusen Wang, Yuling Duan, Yang Zhang

**Affiliations:** Department of Respiratory and Critical Care Medicine, Xingtai People's Hospital, Xingtai 054001, Hebei, China

## Abstract

Air pollution is a primary health threat issue worldwide because it is closely concerned with respiratory diseases. A random survey reported that around 7 million people died because of ambient and household air pollution. Especially, the people suffering from asthma and chronic obstructive pulmonary disease (COPD) are highly affected by air pollutants. The air pollution components induce asthma onset and COPD acute exacerbation, which leads to maximized mortality and morbidity rate. Therefore, the influence of air pollution on COPD should be examined continuously to minimize the mortality rate. Several methods are presented in this field to investigate the relationship between health and pollutants. However, the existing approaches are only predicting the short-term data and have difficulties such as computation time, redundant data in large data analysis, and data continuity. Then, this research introduced the meta-heuristic optimized grey correlation analysis (MH-GCA) to solve the research difficulties. The correlation analysis has several models that identify the relationship between the pollution factors with COPD disease. The method analysis of the particulate matter (〖PM〗_10) in air pollution is more relevant to COPD and lung cancer disease. The grey analysis uses the uncertainty concept to identify the particle influence on air pollution. In the analysis, the cuttlefish optimization algorithm was applied to select more relevant features from the pollutant list that reduces the computation time and correlation analysis rate. The introduced system was evaluated using the air quality dataset and COPD dataset developed with the help of the MATLAB tool. The system increases the influence recognition accuracy (2.48%) and MCC (3.11%) and decreases the error rate (55.89%) for different pollutants.

## 1. Introduction

In 2008, World Health Organization (WHO) reported that 1.3 million people died because of ambient air pollution [1]. The mortality rate has increased to 4.3 million in 2012, and they reported that every year the affected rate increases gradually due to the ambient and household air pollution [2]. Air pollution creates a great impact on the human body and organs; it causes several aggressive diseases [3, 4] such as ischemia heart disease and cardio cerebral vascular disease. In addition to this, pollutants affect the nervous system, urinary system, and digestive system which results in a high mortality rate. Among the various diseases, air pollution influences the respiratory system and creates various diseases like lung cancer, asthma, and chronic pulmonary disease (COPD) [5]. Long-term air pollution is still a major problem worldwide; therefore, air pollutants should be identified to minimize chronic respiratory disease. The components of air pollution varies from one place to another, and they are classified into outdoor and indoor pollutants [6]. The outdoor pollutants such as [7] nitrogen dioxide(*NO*_2_), particulate matter(*PM*), carbon monoxide(*CO*), sulfur dioxide (*SO*_2_) lead (*Pb*), and Ozone (*O*_3_) are creating serious impacts. Therefore, WHO provides the basic guidelines for reducing the impact of these pollutants. These pollutants are received from garbage burning, brush fire, industrial production, transport emission, and forest. The particles that come from these wastes are very small in size, and it has two variants as (*PM*_10_) and(*PM*_2.5_) [8]. According to the air quality indices, *PM*_2.5_ is more dangerous to people's health in most of the countries. The indoor pollutants [9] are the same as outdoor pollutants but the concentration level of indoor pollutants was low. The major reason for this type of pollutants is tobacco smoking, solid fuels, furnishing, poor ventilation, and construction materials. The outdoor pollutants are the main reason for the cardiovascular disease bladder cancer and appendicitis [10]. The higher concentration of the ambient pollutants has maximized the hospitalization and triggered the acute myocardial infarctions. Particle matters are easily traveling via the nanosized central nervous system, which can damage the blood-brain barrier and causes neurodevelopmental disorder, Parkinson's disease, and stroke [11, 12]. Indoor pollutants such as benzene and formaldehyde cause leukemia.

The maximum level of ambient pollution seriously affects COPD patients. Recently, air pollution has highly influenced people's respiratory system. The American Thoracic Society (ATS) [13] reports and provides a guideline about air pollution because most of the respiratory diseases occurred due to pollution. The pollutant's detrimental effects increase the respiratory systems, infection, asthma onset, COPD acute exacerbations, respiratory mortality rate, asthma, and decreased pulmonary functions. COPD is caused by high involvement of air pollutants and creates an inflammatory response in the airway. According to the research, in developing countries, women have a high COPD risk rate because of the smoke exposure while cooking. The particle material pollutants from the fuel combustion leads to lung inflammation and minimize the pulmonary function in COPD patients. High exposure to particle pollution requires hospitalization, emergency care and can even cause death. Although, the WHO and other air pollution control societies give guidelines for avoiding air pollution [14]; important steps are to be taken to control the pollutant levels. Therefore, an air pollutant monitoring system should be incorporated into the field to identify the pollutant level. The pollution monitoring process uses the surrounding and air information to analyze the pollutant impact on the air. The collected air information was analyzed by applying data mining and machine learning techniques [15]. These techniques are performed pre- and post-processing to identify the indoor and outdoor pollutant levels. The traditional systems use only a limited amount of data which means that the system faces difficulties while analyzing a large volume of data [16]. In addition to this, continuity of data should be maintained to improve the overall prediction accuracy. When the system uses a large volume of data, an optimization problem occurs that completely affects the pollutant prediction process. These research problems are overcome by applying the meta-heuristic optimized grey correlation analysis approach. The method uses the fitness function and local and global searching process to investigate each data. From the data characteristics, the correlation between data is identified to predict the influence of air pollutants on COPD disease. Then, the discussed system is implemented using the MATLAB tool, and the effectiveness of the system is evaluated using experimental results and discussion.

Then, the rest of the paper is arranged as follows: Section 2 analyzes the different researchers' work on air pollutant analysis towards the health impact.  Section 3 discusses the working process of introducing meta-heuristic optimized grey correlation analysis based on air pollutant level prediction. The system's effectiveness is evaluated in Section 4, and the conclusion is described in Section 5.

## 2. Related Works

This section describes the detailed review of various researchers' work on air pollutants' impact on human health. Losacco and Perillo [17] discussed the impact of particulate matter on human and animal respiratory systems. The particulate matters are the reason for various diseases such as cardiovascular disease and pulmonary manifestations. According to the research, the size of particles and surface only determines the injury level, biological effect, and oxidative damage. Therefore, this paper analyzes various criteria to resolve the particulate matter impact on air for reducing the mortality rate of both animals and humans.

Soh et al. [18] introduced an adaptive deep learning (ADL) approach to predict air quality. The air pollutants and particulate matters penetrate the body and create several health problems such as respiratory and cardiovascular disease. The author aims to predict air quality with a maximum recognition rate for reducing the mortality rate in the future. This paper uses the Taiwan and Beijing dataset information, which is processed by applying the combination of long-short term memory, convolution, and artificial neural networks. These networks utilize a few hours of meteorological data to predict air quality. The collected data is processed for extracting the terrain information, including the location information, correlation details, and temporal details. This information is fed into the network that predicts the air quality by comparing the pre-trained model. Then, the created system ensures high accuracy by monitoring the air quality for up to 48 hrs.

Guo et al. [19] analyzed the relationship between the sputum inflammatory markers and clinical symptoms along with air pollution in the Beijing area. This work intends to expose the air pollutants that are the main reason for the COPD disease. During this process, data was collected from China Peking University's third hospital. The correlation between the air pollutants and the clinical symptoms was evaluated for 7 days in which different particles were assessed. During the analysis, a COPD assessment test was taken in which particulate matters create the greatest impact on COPD. For this analysis, 78 COPD-infected people and 58 healthy people were considered. The COPD-infected people were isolated from the air pollution for the 7 days of activities in which people's symptoms were gradually reduced.

Ho et al. [20] discussed the chronic obstructive pulmonary disease patient health risk factor due to the air pollution. This work intends to prove that air pollutants create serious issues for pneumonia and COPD-infected patients. The analysis used both normal and COPD-infected people's health details. The patient's information was examined concerning the air pollutant levels to justify the work. From the COPD assessment test, COPD patients were highly at risk while they were inhaling pollutants, especially particulate matters.

Rahi et al. 2021 [21] introduced a firefly-optimized support vector machine (FSVM) for monitoring air quality in smart eHealth systems. This work aimed to predict the air quality for reducing airborne allergies and treatment cost burden. The meteorological data was processed by an introduced monitoring system to improve the outcomes. The data were investigated using the optimization algorithm that selects the most relevant features. Here, the firefly optimized algorithm was utilized for selection purposes. Then, the selected features were processed by a support vector machine that predicts the pollutant index level with 94.4% of accuracy.

Rodríguez-Aguilar et al. [22] recommended the breath print identification process to detect the relationship between COPD and household and smoking air pollution. This work used the Cyranose 320 electronic noses for analyzing the participant's health condition and linked it with the smoking-related air pollution. Here, around 294 participants' information was analyzed by using different methods such as principal component analysis and canonical discriminate analysis. The extracted features were processed with the help of a support vector machine that predicts the breath point with 97.8% of accuracy.

Abugabah et al. [23] applied a meta-heuristic optimized neural network (MONN) for detecting people's lung conditions in urban spaces. The system used the NIH clinical dataset and ELT-COPD information for evaluating people's health conditions. Initially, the min-max normalization process was applied for eliminating the irrelevant data. Then, Hilbert-Schmidt independence criteria were applied to select the optimized features. The derived features are investigated using the optimized classifier that predicts the people's health condition with up to 98.9% of accuracy on the ELT-COPD dataset and 98% on the NIH clinical dataset.

González et al. [24] analyzed the impact of particulate matter 2.4 on labor absenteeism because of COPD in Santiago city. The patient health information was collected from public health authorities which were processed by using Pearson's correlation analysis and mining technique. The correlation analysis determined the relationship between the particulate matter with the COPD risk factor. The concentration level of PM 2.5 level increased gradually, and the patient's health condition was monitored. The report clearly states that COPD people are at high risk when they are inhaling the air with particulate matter.

Khojasteh et al. [25] analyzed the long-term effect of outdoor air pollutants on mortality rate using the non-linear autoregressive neural networks (N-ARNN). This system intended to predict the long-term effects of pollutants on the respiratory problem which was done by using the Dickey–Fuller test. The study was conducted over 9 years, and the data was processed by applying the introduced neural network classifier. The classifier predicted the sensitive pollutants from the collected data. From the analysis, carbon monoxide and nitrogen monoxide created a great impact and lead to an increase in the mortality rate. The introduced network uses the 2-10-1 topology while investigating the inputs. Successful utilization of network functions recognized the pollutants with 0.82% of accuracy and 0.1 error rate value. According to various researchers' opinions, the air pollutants were investigated by applying various machine learning and data mining techniques. Each approach utilized specific functions and templates for detecting pollutant levels. Based on the pollutant level, the impact of health conditions was identified effectively. From various researchers' ideas, this work chose the grey correlation analysis with optimization technique to predict the pollutant level. By utilizing the introduced technique, the following objectives were addressed in this work.

- Improving the pollutant prediction rate by examining the correlation between the features
- Reducing the difficulties while analyzing the large volume of air pollutant data
- Maintaining the system reliability by reducing the optimization problem

## 3. Meta-Heuristic Optimized Grey Correlation Analysis (MH-GCA) of Air Pollutants towards the Pulmonary Diseases

This section discusses the influence of air pollution on pulmonary diseases. The indoor and outdoor air pollutants create a great impact on the respiratory system and cause several diseases such as COPD, asthma, and lung cancer. Among the various diseases, the pulmonary functions have a high risk when the patient inhales the pollutant or particulate matter. Therefore, the air pollutants should be analyzed, and the link between the pollutants and infection had to be predicted to reduce the mortality rate. The relationship between the particles and people's health was analyzed by applying the correlation analysis process. The pollutant characteristics and involvement were identified with the help of the air quality index and monitoring criteria. In addition to this, patient's pulmonary disease details was required for improving the overall performance of the study. The overall working process of MH-GCA based air pollution influence on COPD is illustrated in Figure 1.

### 3.1. Materials Collection

This section discusses the dataset utilized in this work to analyze the influence of air pollutants on pulmonary disease. Here, air quality data in India (2015–2020) Kaggle dataset [26] were utilized for investigating air pollutants. The dataset has hourly-based collected information and the air quality index (AQI) of various stations in India. The air quality and monitoring process are more important in analyzing people's health. The dataset consists of AQI and air quality data which were collected daily and hourly based in India's several cities. A detailed discussion of AQI computations is discussed in Section 3.2. The dataset has almost India's top most popular cities such as Chennai, Amaravati, Ahmedabad, Bengaluru, Amritsar, Aizawl, Chandigarh, Brajrajnagar, Kochi, Hyderabad, Ernakulam, Coimbatore, Thiruvananthapuram, Delhi, Kolkata, Patna, Lucknow, Visakhapatnam, Talcher, Shillong, and Mumbai. Here, a few air pollutant data are shown in Table 1.

Along with the air quality dataset, the pulmonary infection disease dataset needs to be collected for evaluating the influence of air pollutants on disease. Then, COPD patients' dataset [26] was utilized, which was collected from Kaggle that used to identify the information about the pulmonary patients. COPD is one of the progressive lung diseases which is most common with the chronic bronchitis and emphysema. Most of the COPD-affected people were influenced by these two conditions; the emphysema silently affects the air sacs present in the lungs and interferes with the outward airflow. Bronchitis affects the narrowing and inflammation of the bronchial tubes. The dataset consists of 101 patients' information with 24 variables. The information were gathered according to the comorbidities and disease severity. In addition to this, the details were collected based on the anxiety, quality of life, depression, and walking ability. According to the discussion, different information was collected, and the sample details are illustrated in Figure 2.

After collecting dataset information, the link between the air pollutant data and COPD disease should be analyzed for reducing the mortality rate. To achieve the objective of the system, initially, the air quality index (AQI) should be computed for observed data. From the computed AQI value, the relationship between the health data was investigated using the optimized grey correlation analysis approach.

### 3.2. Methods Analysis

#### 3.2.1. Air Quality Index Computation

The air quality standard or index (AQI) is announced by the environment protection law of the China Republic and atmospheric pollution prevention control of the China Republic. The AQI helps to measure the air quality standard in the short term that is used to measure the pollutant concentration level. The recorded concentration level not only determines the air quality but also measured the air pollution. The air pollution index is computed for almost every outdoor pollutants such as nitrogen dioxide (*NO*_2_), particulate matter (*PM*), carbon monoxide (*CO*), sulfur dioxide (*SO*_2_) lead (*Pb*), and Ozone(*O*_3_). The pollutant concentration ranges belong to *C*_*i*,*j*_ ≤ *C*_*i*_ ≤ *C*_*i*,*j*+1_. Then, the AQI value is estimated using

(1) $$\begin{array}{c} I_{i}=\frac{\left(C_{i}-C_{i,j}\right)\left(I_{i,j+1}-I_{i,j}\right)}{\left(C_{i,j+1}-C_{i,j}\right)}+I_{i,j}\text{.} \end{array}$$

In (1), pollutant *i* related index, the concentration level of *i*th pollutant is denoted as*C*_*i*_, *ith* and pollutant changed into the *jth* index level is represented as*I*_*i*,*j*_. According to (1), each pollutant index value is calculated from the pollutant concentration level and computed values are arranged in sorting order. The maximum index value is selected as the AQI value which is represented as

(2) $$\begin{array}{c} AQI=\max\;\left\{I_{1},I_{2},I_{3}\ldots \ldots I_{n}\right\}\text{.} \end{array}$$

The environment is continuously influenced by air pollution; therefore, the state council reviewed air quality standards according to the environmental science research report. The AQI values are more important to determine the air quality, and it is the representation of the atmospheric conditions. Therefore, the index value should be computed by considering the individual pollutants such as(*O*_3_,(*CO*),(*SO*_2_), (*PM*), (*NO*_2_), and(*Pb*). Then, IAQI value is estimated using

(3) $$\begin{array}{c} {IAQI}_{P}=\frac{{IAQI}_{H}-{IAQI}_{L}}{{BP}_{H}-{BP}_{L}}\left(C_{P}-{BP}_{L}\right)+IAQI\text{.} \end{array}$$

The (3) was utilized to review the air quality standard computation; pollutant P air quality index is defined as *IAQI*_*P*_; P concentration value is represented as *C*_*P*_; concentration breakpoint is *BP*_*H*_, which is not more than the *C*_*P*_; concentration breakpoint *BP*_*L*_, which is not less than the *C*_*P*_. *BP*_*H*_ and *BP*_*L*_ *the*related index was measured as *IAQI*_*H*_ an d *IAQI*_*L*_. The computed individual pollutant index values are arranged in the sorting order to get the revised AQI value.

(4) $$\begin{array}{c} AQI=\max\;\left\{{IAQI}_{1},IAQI_{2},IAQI_{3}\ldots \ldots {IAQI}_{n}\right\}\text{.} \end{array}$$

According to the above discussion, the AQI values are computed for collected air quality dataset information. Here, Thiruvananthapuram city information was collected because it has two stations that are used to compare the air pollutant level effectively. Here, hourly-based collected information was utilized to evaluate the pollutant level in a specific area. Then, the graphical analysis of the AQI computation is illustrated in Figure 3.

Figure 3 illustrates the air quality index computation for the air quality dataset information. The pollutants were analyzed in 24 hrs and 8 hrs to estimate the concentration level. The AQI values were estimated for seven pollutants such as O_3_, CO, NOx, SO_2_, PM_10_, and PM_2.5_. The CO and O_3_ are collected for the last 24 hrs. After that, each pollutant measure was converted to a sub-index value according to pre-defined groups. From the computation, the maximum sub-index value was selected as the AQI value; here, at least one pollutant should be considered to compute the value else three pollutants should be presented. The severity of the pollutants was estimated based on the AQI value, and the impact of the pollutants is illustrated in Table 2 [27].

Table 2 clearly states the impact of the pollutants on the people, which is measured by using the AQI value. The AQI analysis clearly shows that most of the pollutants cause respiratory problems such as asthma, COPD, and lung cancer. However, there is no significant evidence to prove the relationship between air pollutants and COPD problems. Therefore, this research study focuses on the correlation analysis for investigating the influence of air pollutants on COPD disease.

#### 3.2.2. Grey Correlation Analysis

Grey correlation analysis is a measure for identifying the degree of association between the data by grey relational grades. The correlation analysis can process a small amount of data, is easier to process, and the results are more understandable and intuitionistic. However, this method requires an effective training model to process a large volume of data. The training model used a set of pre-defined features with labels that were used to predict the exact relationship between data. In the correlation analysis, the similarity between the sequences of data was compared with the training pattern for assessing the relationship. Generally, the particulate matters are more correlated with lung disease (i.e., COPD) compared to the other pollutants such as SO_2_, NO_2_, and CO. Therefore, an effective correlation analysis should be performed to determine the exact relationship between the data. Initially, the comparison and reference sequence of data should be defined. The sequence of data represents the characteristics of the reference information; therefore, the changes in the data sequence affect the behavior of the reference sequence. That is, the air quality data represents the people's health characteristics; the changes in the air quality influence the people's health. Considerd, *X*_0_=[*x*_0_(1), *x*_0_(2), *x*_0_(3),……*x*_0_(*n*)] is the reference data and *X*_*i*_=[*x*_*i*_(1), *x*_*i*_(2), *x*_*i*_(3),……*x*_*i*_(*m*)] is comparison data. After that, the non-dimensional method has to be applied to the comparison and reference data. The non-dimensional data analysis approach minimizes the difficulties in the factor analysis process. Each data has different factors that are difficult to determine while comparing the reference and comparison data. Therefore, the non-dimensional-based normalization process applied to the data is shown in equation as follows:

(5) $$\begin{array}{c} X_{0}\left(j\right)=\frac{x_{0}\left(j\right)-x_{0,\min}}{x_{0,\max}-x_{0,\min}}\text{.} \end{array}$$

In (5), the reference sample serial number is *j*, reference sequence maximum value is denoted as *x*_0,max_, reference sequence minimum value is *x*_0,min_. This process is further applied to the comparison sequence that is defined as

(6) $$\begin{array}{c} X_{ij}=\frac{x_{ij}-x_{ij,\min}}{x_{ij,\max}-x_{ij,\min}}\left(1\leq j\leq m,i\leq j\leq n\right)\text{.} \end{array}$$

In (6), the comparison sample ith factor, the jth sample is denoted as *X*_*ij*_, the maximum value of the comparison sample is *x*_*ij*,max_ and minimum value is *x*_*ij*,min_. After normalizing the data, the correlation between the sequences was computed. The degree of correlation values varied from one pollutant to another. Then, the correlation *ζ*(*X*_*i*_) between two sequences were estimated.

(7) $$\begin{array}{c} \xi_{i,1}\left(j\right)=\frac{\min_{i}\min_{j}\left|x_{0}\left(j\right)-x_{ij}\right|}{\left|x_{0}\left(j\right)-x_{ij}\right|+\rho \max_{i}\max_{j}\left|x_{0}\left(j\right)-x_{ij}\right|}\text{,}\\ \xi_{i,2}\left(j\right)=\frac{\max_{i}\max_{j}\left|x_{0}\left(j\right)-x_{ij}\right|}{\left|x_{0}\left(j\right)-x_{ij}\right|+\rho \max_{i}\max_{j}\left|x_{0}\left(j\right)-x_{ij}\right|}\text{.} \end{array}$$

After computing the *ξ*_*i*,1_(*j*) and *ξ*_*i*,2_(*j*), the resolution coefficient was estimated as *ζ*_*i*_(*j*)=*ξ*_*i*,1_(*j*)+*ξ*_*i*,2_(*j*). Finally, the degree of correlation *γ*_*i*_was estimated from the *ζ*_*i*_(*j*) the value which was done by using

(8) $$\begin{array}{c} \gamma_{i}=\frac{1}{n}\overset{n}{\underset{j=1}{\sum }}\zeta_{i}\left(j\right)\left(i=1,2,\ldots .m\right)\text{.} \end{array}$$

The computed *γ*_*i*_ value is related to both reference and comparison sequence in different situations. The *γ*_*i*_ value was measured continuously because it was changed frequently; therefore, it was predicted at every curve point for identifying the relationship between the reference and comparison sequence. The computed *γ*_*i*_ values were sorted to get the correlation between the data effectively.

#### 3.2.3. Learning Model

Here, the comparison sequence was generated with the help of the optimized neural model. The back propagation neural model (backdrop) was utilized to create the template or comparison sequence for the data for solving the large data computation issue. The backdrop algorithm was effectively utilized for training the network and improving the overall relationship prediction accuracy. The algorithm used the network inputs and parameters (weights and bias) values for calculating the output. The backdrop algorithm estimated the network gradient value and computed the loss function while analyzing inputs-output. The algorithm propagated the error value to previous layers and updated network parameters to minimize the loss value. During this process, the chain rules were applied for making successful network updating. The backdrop algorithm calculated the weight value depending on the loss function. Consider that *x* is the input vector, *y* is the output which obtains the value as (0, 1), *C* is loss function (cross-entropy), number of layers in the network is *L*, *l* and *l* − 1 layer weight values are represented as *W*^*l*^, and the activation function is *f*^*l*^ (SoftMax). According to these parameters, the combination of network performance is illustrated in equation as follows:

(9) $$\begin{array}{c} g\left(x\right)=f^{l}\left(W^{L}f^{l-1}\left(W^{L-1}\ldots ..f^{1}\left(W^{1}x\right)\ldots \text{.}\right)\right)\text{.} \end{array}$$

By using (9), output *y* was computed for every input *x* in the training model. During this process, the loss function was estimated for *g*(*x*) which is defined as *C*(*y*_*i*_, *g*(*x*_*i*_)). The model used the fox optimization algorithm to update the network parameter. The optimization algorithm reduces the continuous and discrete optimization problem. The algorithm has two phases such as exploration searching (global search) and prey moving (local search). The optimal network parameters were selected at *t* iteration from a number of parameters such as $\bar{a}=\left\{a_{1},a_{2},\ldots \ldots a_{n}\right\}$. For specific parameter or fox at *t* is denoted as ${\left({\bar{a}}_{j}^{i}\right)}^{t}\text{.}$ Each fox moving in the search spaced to identify the optimal solution according to the fitness function $f{\left({\bar{a}}_{j}^{i}\right)}^{t}\in {\mathbb{R}}^{n}$. During the computation, parameters *b*, *c* ∈ *ℝ* is utilized. Then, the global searching process was performed to identify the best features. The fox searches for their food and conveys its message to the herd to make the exploration search. The global search used the Euclidean distance measure to compute the difference between two parameters defined as

(10) $$\begin{array}{c} d\left({\left({\bar{a}}^{i}\right)}^{t},{\left({\bar{a}}^{best}\right)}^{t}\right)=\sqrt{\left\|{\left({\bar{a}}^{i}\right)}^{t}-{\left({\bar{a}}^{best}\right)}^{t}\right\|}\text{.} \end{array}$$

Each fox moves on the search space, the best solution is identified, and the identification of a specific fox is defined as

(11) $$\begin{array}{c} {\left({\bar{a}}^{i}\right)}^{t}={\left({\bar{a}}^{i}\right)}^{t}+\alpha sign\left({\left({\bar{a}}^{best}\right)}^{t}-\left({\bar{a}}^{i}\right)\right)\text{.} \end{array}$$

The searching process uses the scaling parameter; $\alpha \in \left(0|,|d|\left({\left({\bar{a}}^{i}\right)}^{t},{\left({\bar{a}}^{best}\right)}^{t}\right)\right.$ which was selected in every iteration. After every iteration, the fox position was updated with the family members for improving the searching process. After identifying the food, the fox moved the prey without creating any disturbance. Then, the attacks were performed and movement was determined using the random value *μ* ∈ (0,1). The value only decided the movement of prey in search space.

(12) $$\begin{array}{c} \left\{\begin{array}{cc} move\;closer\text{,} & if\mu >0.75\text{,}\\ stay\;and\;disguise\text{,} & if\mu \leq 0.75\text{.} \end{array}\right. \end{array}$$

The random value used the scaling parameter *a* ∈ (0, 0.2) and observation angle (∅_0_ ∈ (0,2*π*)) to determine the food or parameter. Then, the radius value (*r*) was computed to attack the food defined as

(13) $$\begin{array}{c} r=\left\{\begin{array}{cc} a\frac{\sin\left(\emptyset_{0}\right)}{\emptyset_{0}}, & if\emptyset_{0}\neq 0\text{,}\\ \theta \text{,} & if\emptyset_{0}=0\text{.} \end{array}\right. \end{array}$$

By considering these parameters, the fox food searching process was updated with angler value and scaling parameter defined as

(14) $$\begin{array}{c} \left\{\begin{array}{c} a_{0}^{new}=br.\;\cos\left(\emptyset_{1}\right)+a_{0}^{actual}\text{,}\\ a_{1}^{new}=br.\;\sin\left(\emptyset_{1}\right)br.\;\cos\left(\emptyset_{2}\right)+a_{1}^{actual}\text{,}\\ \ldots \ldots ..\\ a_{n-1}^{new}=br.\;\sin\left(\emptyset_{1}\right)br.\;\sin\left(\emptyset_{2}\right)+\ldots \ldots .+br\;\sin\;\left({\emptyset_{n-1}+a}_{n-1}^{actual}\right)\text{.} \end{array}\right. \end{array}$$

Then, the fox performed operations such as reproduction or leaving the herd. Here, the fitness function was utilized to determine the worst/best fitness value, and the fitness function was computed as fit=∑_*k*=0_^individual^|*f*(*x*^*k*^) − *f*(*x*^ideal^)|/individuals. According to the fitness value, two individuals were selected as alpha couple which helped to determine the habitat center value${\left({habitat}^{\left(center\right)}\right)}^{t}={\left({\bar{x}}^{\left(1\right)}\right)}^{t}+{\left({\bar{x}}^{\left(2\right)}\right)}^{t}/2$. Then, the distance between the alpha couple and habitat center was computed as $\sqrt{\left\|{\left({\bar{x}}^{\left(1\right)}\right)}^{t}-{\left({\bar{x}}^{\left(2\right)}\right)}^{t}\right\|}$ . Based on the computation, the replacement process was performed using the following condition:

(15) $$\begin{array}{c} \left\{\begin{array}{cc} new\;individual\text{,} & ifk\geq 0.45\text{,}\\ reproduction\;of\;alpha\;couple, & ifk<0.45\text{.} \end{array}\right. \end{array}$$

Then, the new individuals were generated as $k{\left({\bar{x}}^{\left(1\right)}\right)}^{t}+{\left({\bar{x}}^{\left(2\right)}\right)}^{t}/2;k\in \left(0,1\right)$ and again the searching process was performed to get a better value.

The searching process used the different parameters and fitness functions to estimate the optimized value from the set of values. The selected parameters were applied to the neural model to update the network parameters. This process helped to reduce the loss function and improves the prediction accuracy. The generated template inputs were treated as a comparison sequence utilized to predict the correlation between the air quality data and disease. Then, the association of air quality influence on COPD is discussed in the results section.

## 4. Experimental Results and Analysis

This section evaluates the effectiveness of the introduced optimized grey correlation analysis based on air quality influence on people's health conditions is analyzed. The discussed system's effectiveness was evaluated using the air quality dataset and COPD datasets which were collected from the Kaggle database. The air quality dataset consists of pollutants information that was collected in terms an hourly and daily basis. The gathered details were analyzed using air quality index (AQI) computation for getting the concentration and air quality information. Then, the COPD dataset consists of a set of information that belongs to the lung cancer characteristics. In addition to this, general statistical reports were taken to investigate the number of lung cancer patients. According to the clinical report, the number of lung cancer patients is increasing year by year. The females are highly influenced by the lung disease compared to the males which directly indicates that non-smoking people are highly influenced by lung diseases like lung cancer and COPD.

### 4.1. Correlation Analysis with the COPD

This section analyzes the influence of air pollution on lung infection called pulmonary disease (COPD). The correlation investigation used the reference sequence and comparison sequences to predict the influence of air pollution. The collected COPD dataset information was processed by the fox optimized backprop neural model that generates the template for the features. The created templates were considered as the reference sequence and computed AQI values were treated as comparison sequences. The influence of air pollution varied from time to time which may cause COPD in various time lags. Therefore, the analysis considered different time lags for making the correlation analysis. The association analysis clearly shows that indoor and outdoor air pollution was highly correlated with COPD disease. According to the study, the people infected by COPD have 10 *μ*g/m^3^ high in PM_10_ daily consumption. According to a study on air pollution, people who inhaled 50 *μ*g/m^3^ of SO_2_, suspended particulates, black smoke, O_3_, and NO_2_ are highly prone to COPD.The infected people were continuously observed; they were having 1.02 (0.98 to 1.06) of black smoke, 1.04 (1.01 to 1.06) of suspended particulates, 1.02 (1 to 1.05) of NO_2,_ and 1.04 (1.02 to 1.07) of O_3_. The conception of these pollutants was increased day by day which led to severe health issues. Then, the incidence of air pollutants with COPD [26] is illustrated in Table 3.

Table 3 illustrates the air pollutant incidence influence on the COPD disease out of which particulate matter (PM) had a high influence on the COPD compared to other pollutants. The pollutant influence was investigated from the relative risk (RR) rate of 2.5%, which is higher comparatively. Then, O_3_ and PM_2.5_ were the next influencing pollutants that had 1.04% and 1.03% of RR. Then, NO_2_, SO_2_, and TSP (total suspended particles) had 1.02% of RR in COPD disease. These pollutant influences were investigated on time/lag of 0 to 5. Then, the graphical representation of pollutants versus concentration level and pollutants versus RR is illustrated in Figures 4(a) and 4(b).

Figure 4(a) clearly states that the particulate matter (PM) and ozone (O_3_) had highly influenced the COPD patient up to 22.22% compared to the other pollutants such as NO_2_ (11.11%), SO_2_ (11.11%), and TSP (11.11%). The high concentration level indicates that the air has poor quality, and it leads to severe health problems. The concentration level is computed from the AQI, and the characteristics of the air are illustrated in Table 2. Once the concentration level is high, then, the respective risk rate (RR) is also high. From Figure 4(b), the particulate matter has a 32.77% risk rate compared to other pollutants NO_2_ (13.37%), O_3_ (13.63%), SO_2_ (13.37%), and TSP (13.37%) to the 95% of confidence interval (CI). In addition to this, the effectiveness of the system is further evaluated with accuracy, Matthew's correlation analysis, and error rate value.

The discussed optimized grey correlation analysis used the neural model to train the comparison sequence which helps to improve the overall air quality influence prediction rate. Moreover, this method was used to solve the misclassification error rate and optimization problem. The comparison sequence was generated by applying the sequence of data to the different layers. The network used the input, weight, bias, and activation function to estimate the output value. The outputs were more likely to utilize the comparison with the reference sequence. Depending on the comparison, the air quality index was predicted effectively. The pollutant levels were examined every day, but for the period of COPD, the lags were considered to identify the best result. Then, the obtained accuracy results for pollutant and different period was compared (Figures 5(a) and 5(b)).

Figure 5(a) illustrates the accuracy analysis of the air pollution prediction towards the COPD disease. Here, the analysis was performed with different pollutants, and the introduced meta-heuristic optimized grey correlation analysis (MH-GCA) predicted the pollutants effectively compared with the adaptive deep learning (ADL) [28], firefly optimized support vector machine (FSVM) [29], meta-heuristic optimized neural network (MONN) and non-linear autoregressive neural networks (N-ARNN). The introduced method used the backprop layer functions such as *C* and *f*^*l*^ for every input*x*. The network layer used the weight *W*^*l*^ and bias *b* value for computing the output *y* using the *f*^*l*^ activation function. Then, the output layer combined the output of every layer and got the net output value *g*(*x*). These layers used the COPD dataset, and characteristics were input and produce the output which was the severity of the disease. Once the people were affected by COPD, their surrounding air quality was examined, and obtained details were captured to create the comparison sequence. The effective way of obtaining details helped to improve the accuracy while matching the reference and comparison sequence. The introduced method also predicted the pollutant influence on COPD at various time-intervals with high accuracy (Figure 5(b)). In addition to the accuracy value, the correlation between the air pollutant and COPD was examined effectively. The efficiency was evaluated on different pollutants and various time intervals and results are illustrated in Figures 6(a) and 6(b).

Figure 6 depicts the correlation analysis of the introduced MH-GCA approach on different pollutants and day interval. Here, the method utilized the non-dimensional method for normalizing the collected air quality data which simplified the correlation analysis. During the process, minimum *x*_0,min_ and maximum *x*_0,max_ values were utilized to predict the normalized value for both reference and comparison sequence. The normalization process changed the attributes in a simplified and similar manner that reduced the overall difficulties in the comparison process. After that, correlation *ζ*(*X*_*i*_) and degree of correlations *γ*_*i*_ were computed to identify the air quality influence. Once the air quality information was collected from the COPD patient life area, the respective AQI value was computed for each pollutant defined in (2) and (4). The computed AQI value is shown in Table 2 for predicting the particular area characteristics. Depending on the computation, the introduced approach effectively predicted the air pollution of COPD people. During the analysis, the system used the fox optimization algorithm for updating the learning model that minimized the deviation between the actual and predicted value. The effectiveness of the system was further evaluated using the error rate. Then, the obtained results are shown in Figures 7(a) and 7(b).

Figure 7 illustrates the error rate analysis of various pollutants and day intervals while investigating the pollutants on COPD. The neural model was utilized for training the COPD patient with relevant air quality information. The model generated the comparison sequence for inputs during the process, and network parameters were updated for minimizing the loss of function C. The optimization method used the as fit=∑_*k*=0_^individual^|*f*(*x*^*k*^) − *f*(*x*^ideal^)|/individuals value for identifying the best parameter in the search space. The searching process used local and global search to predict the optimized solution. The best solution was predicted with the help of the distance measure that identified the most relevant feature from the search space. Then, the scaling parameter and radius values were utilized to predict the new individual in the search space which helped to update the network parameter effectively. The optimized method network parameter updating procedure minimized the deviation between actual and predicted value. The overall results are summarized in Tables 4 and 5.

## 5. Conclusion

Thus, the paper analyzes the meta-heuristic optimized grey correlation analysis (MH-GCA) based on air pollution influence on COPD. Initially, the air quality dataset and COPD dataset were collected from the Kaggle database. For air pollution information, AQI values were computed for each and combination of three pollutants. According to the pollutant values, the concentration levels were computed for comparing the sequence. Then, the comparison sequence related templates were created with the help of the backprop algorithm. The learning model used the SoftMax activation function to predict the output value. Then, the fox optimization food searching process and reproduction procedure were applied for updating the network parameter. The effective food searching process minimized the deviation error. The generated neural model patterns were compared with the reference pattern for identifying the influence of the air pollution on COPD. The influence was investigated using the correlation analysis approach which used the degree of correlation and correlation coefficient. Thus, the introduced MH-GCA approach recognized the air pollutant influence on COPD with 2.48% accuracy, 3.11% of MCC, and minimum error rate (55.89%) on different pollutants compared to other methods. Thus, the introduced system resolved the research problem by successful examination of AQI and correlation value. In the future, the system performance will be improved for analyzing the huge volume of data with maximum prediction accuracy.

## Figures and Tables

**Figure 1:** Working structure of meta-heuristic optimized grey correlation analysis (MH-GCA).

**Figure 2:** Sample data of COPD dataset.

**Figure 3:** AQI computation for air quality dataset information.

**Figure 4:** (a) Pollutants vs. concentration level and (b) pollutant vs. RR.

**Figure 5:** Accuracy (a) different pollutants (b) day interval.

**Figure 6:** MCC (a) different pollutants (b) day interval.

**Figure 7:** Error rate analysis of (a) different pollutants (b) day interval.

**Table 1:** Sample air quality dataset.

Station ID	Date	PM_2.5_	PM_10_	NO	NO_2_	NOx	NH_3_	CO	SO_2_	O_3_	Benzene	Toluene	Xylene	AQI
AP001	^########^	71.36	115.75	1.75	20.65	12.4	12.19	0.1	10.76	109.26	0.17	5.92	0.1	
AP001	^########^	81.4	124.5	1.44	20.5	12.08	10.72	0.12	15.24	127.09	0.2	6.5	0.06	184
DL030	5/2/2018	91.93	162.07	40.6	41.8	82.39		0.35		44.66	0	0	0	178
DL030	5/3/2018	0.66	51.85	10.69	37.61	48.29		0.47		15.18	0	0	0	186
GJ001	^########^	96.71		19.89	101.08	64.15		19.89	127.91	54.97	22.98	101.88	17.71	650
GJ001	^########^	75.14		29.6	89.68	65.84		29.6	116.39	67.14	19.73	87.41	17.33	515
HR011	2/9/2018	246.01	401.91	113.05	11.23	124.28		2.62		3.64				377
HR011	^########^	164.11	273.52	109.38	14.29	123.67		2.63		3.53				358
HR013	4/1/2020	31.34	53.55			0		0.54	24.62	50.56	3.6	7.44	14.32	76
HR013	4/2/2020	25.67	46.97			0		0.53	25.33	62.02	0	0	0	74
HR014	8/3/2016	30.94		2.99	5.01	7		0.37	1.86					
HR014	8/4/2016	29.94		3.01	4.93	6.99		0.31	1.94					52
HR014	8/5/2016	29.33		3.23	4.35	6.91		0.41	1.76					46
AP001	^########^	117.46	181.64	4.26	41.1	25.32	17.34	0.13	28.79	94.63	0.36	6.21	0.17	252

**Table 2:** Impact of the pollutant levels.

S. no	AQI level	Characteristics	Impact
1	0 to 50	Good	Minimum impact
2	51 to 100	Satisfactory	Minor breathing discomfort for sensitive people
3	101 to 200	Moderate	Lung, heart disease people, children, and older adults feel discomfort while breathing
4	201 to 200	Poor	Prolong exposure to the pollutant causes the breathing discomfort
5	301 to 400	Very poor	Prolong exposure causes respiratory illness
6	>400	Severe	The respiratory problem occurs to people even healthy people

**Table 3:** Air pollutant incidence towards COPD.

S. no	Pollutants	Pollutants concentration	*RR* (%)	CI of 95%	Lag
1	NO_2_	50 *μ*g/m^3^	1.02	1.00 to 1.05	1 to 3
2	O_3_	10 *μ*g/m^3^	1.04	1.02 to 1.07	1 to 3
3	PM_10_	10 *μ*g/m^3^	2.5	0.93 to 3.3	0 to 5
4	PM_2.5_	10 *μ*g/m^3^	1.03	1.03 to 1.04	0.5
5	SO_2_	50 *μ*g/m^3^	1.02	0.98 to 1.06	1 to 3
6	TSP	50 *μ*g/m^3^	1.02	1.00 to 1.05	1 to 3

**Table 4:** Summary of air pollution influence on COPD for different pollutants.

Metrics	ADL	FSVM	MONN	N-ARNN	MH-GCA	Findings (%)
Accuracy	94.57	96.72	96.14	96.83	98.45	2.48
MCC	0.953	0.974	0.962	0.974	0.992	3.11
Error rate	0.231	0.2065	0.1843	0.157	0.086	55.89

Inference: the introduced MH-GCA approach increased recognition of the air pollutants influence on COPD with 2.48% of accuracy, 3.11% of MCC and minimized the deviation up to 55.89% for various pollutants.

**Table 5:** Summary of air pollution influence on COPD for different day interval.

Metrics	ADL	FSVM	MONN	N-ARNN	MH-GCA	Findings (%)
Accuracy	94.503	96.611	95.862	97.248	98.647	2.69
Error rate	0.949	0.96422	0.95963	0.96762	0.99488	3.125
MCC	0.22831	0.20795	0.18383	0.15586	0.0869	54.97

Inference: the introduced MH-GCA approach increased recognition of the air pollutants influence on COPD with 2.69% of accuracy, 3.125% of MCC and minimized the deviation up to 54.97% for different day intervals. Thus, the introduced MH-GCA approach successfully predicted the air pollutant influence on COPD compared to other methods. Therefore, the COPD-infected people were aware of the pollutants and managing their health condition according to the situation. In addition to this, normal and COPD-infected people can forecast the daily air pollution via any freely available app and avoiding outdoor activities.

## Data Availability

No data were used to support this study.
